This article has been retracted.

# The Design of Psychological Education Intervention System in Universities Based on Deep Learning

**DOI:** 10.1155/2022/9208172

**Published:** 2022-06-03

**Authors:** Yuefen Wang, Dianyi Yang

**Affiliations:** School of Marxism, Northeast Forestry University, Harbin, Heilongjiang 150040, China

## Abstract

With the rapid development of Chinese society and economy as well as the deepening of the reform of the higher education management system and the change of employment mode of graduates, college students face various challenges of frustration and pressure in the areas of value and ethical concepts, interpersonal relationships, behavior, life, and employment. Some students who are relatively fragile psychologically are unable to bear the heavy pressure of frustration and challenges, and are prone to psychological crisis, overreacting, and even hurting others or self-injury or suicide. How to solve the current psychological problems of college students and help them become adults and talents is a new task and a serious challenge for college students' mental health education under the new situation. With the development of the Internet, more and more people are expressing their emotions in social networks, including suicidal intentions, which creates new opportunities for suicide prevention. If suicide risk can be automatically identified using microblogs, it can open up new directions for suicide prevention efforts. This paper is based on the use of deep learning to build a social media suicide identifier to explore the possibility of assessing individual users' suicide in real time through social platforms. To verify the effectiveness of this algorithmic model, the keyword attributes used by the algorithm are statistically analyzed and compared with the prediction results of two other algorithmic models. The experimental results show that the algorithmic model based on deep learning can be more effective in predicting the suicide risk of microblog users.

## 1. Introduction

College students, as a special social group, are in a period of dramatic changes in their physical and mental development. Facing various changes in society, environment, and themselves, they are prone to changes in ethics, cognitive patterns, behaviors, personality traits, values, interpersonal relationships, employment concepts, etc., which can easily lead to psychological imbalance and psychological crisis [1].

At present, the issue of psychological crisis and crisis intervention among college students is getting more and more attention from colleges and universities, and many schools have offered mental health education courses and set up special counseling and guidance centers. This is both the result of higher education reform and the inevitable trend of positive psychology development [2].

A study shows that in the mid-1980s, 23.25% of college students in China had different degrees of psychological disorders, which rose to 25% in the 1990s, and in recent years, college students with the tendency of psychological disorders accounted for 20%–30% of the total number of college students. According to incomplete statistics, the prevalence of psychological disorders among college students in China is above 16%, and 50% of college students are in a subhealthy or unhealthy state [3]. The issue of mental health education for college students has attracted great attention from the society.

For this reason, the state has introduced a series of policies to guide and help college students to solve their psychological problems. At present, all colleges and universities in China have added mental health education courses as compulsory courses; psychological files are established for new students to detect students with psychological disorders in a timely manner [4]. This reflects an important factor that the psychological crisis intervention system for college students is not perfect. Therefore, colleges and universities should provide a perfect service system and guarantee system for college students' psychological health, and at the same time, families and society should also actively participate in the intervention system for college students' psychological crisis in some ways to help them overcome the crisis and grow up to be successful [5].

In recent years, colleges and universities have begun to pay special attention to the psychological crisis and crisis intervention of college students, and many of them try to establish a comprehensive and multilevel psychological crisis intervention system. However, from the current situation of domestic research, most of the domestic research on psychological crisis intervention for college students is limited to the study of institutions, teams, methods, and means on college campuses, and the establishment of a standardized and professional psychological crisis intervention system in many colleges and universities is still at the stage of thinking and research, without establishing a complete theory of psychological crisis intervention system. This is far from the mental health condition of college students and the needs of mental health education in colleges and universities [6]. Establishing a set of scientific psychological crisis intervention system on this basis is of great theoretical significance to improve the level of organization and intervention of psychological crisis of college students in universities and raise it to the level of defense.

On the other hand, the domestic and foreign research literature on the description of Marxist theory on the comprehensive development of human being and the relationship between human being and society is not thorough enough and not very closely integrated, thus causing the guidance of Marxist theory on the mental health of college students to be greatly reduced. The guiding effect of Marxist theory on college students' mental health is greatly reduced. In addition, the research on the psychological crisis of college students in China is mostly based on foreign theories [7]. This study will try to make the theory and practice of psychological crisis intervention more suitable for China's national conditions and promote the localization of psychological crisis intervention research in China. This study will try to make the theory and practice of psychological crisis intervention more suitable for our country and promote the localization of psychological crisis intervention research in China [8].

## 2. Related Work

Western research on psychological crisis theory originated in the first half of the twentieth century in the United States, the Netherlands, and other countries. Reference [9] proposed a more comprehensive developmental model. That is, precrisis equilibrium state, crisis generation, and postcrisis equilibrium state; precrisis equilibrium state is a stable state between individuals using daily coping methods and problem-solving skills to maintain the environment; [10] takes college students as the research object and focuses on describing the establishment of a psychological crisis intervention system for college students, focusing on college students' psychological crisis-prone population, psychological crisis prevention and suicide expectation, and college students' psychological crisis social support system of college students; [11] proposed the construction of a college students' psychological crisis intervention system consisting of six-in-one, including a crisis prevention subsystem, a four-way interactive crisis warning subsystem, and a five-level linked crisis intervention subsystem; [12] proposed the construction of a college students' psychological crisis intervention system by combining the basic features of the system and analyzed the feasibility and effectiveness of the system; [13] looked at the institutions, mechanism, system as well as preventive education and professional intervention on the construction of psychological crisis intervention system for college students; [14] takes positive psychology and ecosystem theory as the starting point and proposes to construct a three-dimensional ecosystem of psychological crisis intervention for college students, which takes school-family-society as the horizontal section and four stages of preventive education, early warning, crisis intervention, and posttracking as the vertical section; [15] proposes to build a comprehensive three-dimensional psychological crisis prevention and intervention system of individual-family-school-society, which should start from the whole perspective of crisis warning, crisis assessment, crisis intervention, and postcrisis intervention; [16] believes that we should integrate the existing mental health education resources of colleges and universities, strive to improve the psychological quality of students, build a system that focuses on the psychological health of all students as the fundamental, with convenient psychological counseling as the main direction. The mechanism of psychological crisis intervention for college students, which is based on in-depth interviews with college students, [17] proposes to try to build a network system of psychological crisis intervention for college students from four perspectives of crisis intervention: early warning, defense, stress, and operation with the development of technology and network so as to ensure the timely and effective psychological crisis intervention for college students [18] and believes that according to “human being is the sum of all social relations,” the orderly psychological crisis intervention system should be built. According to “human being is the sum of all social relations,” it is believed that orderly social support has a significant positive effect on the physical and mental health of college students, and it is believed that providing strong social support to college students in crisis is the focus of psychological crisis intervention for college students.

From the above studies, it can be seen that the current domestic research on college students' crisis intervention is mainly distributed in the fields of sociology, psychology, education, medicine, and management [19]. In terms of research methods and forms, most of them use the literature research method, and discursive research is the main part, while argumentative practice is rare. The empirical research mainly investigates the personality and psychological characteristics of college students, the crisis events that have occurred, the way of coping with the crisis, and the current situation of social support. In terms of theories based on research, domestic research involves theories such as crisis prevention theory, crisis early warning theory, crisis intervention theory, stress intervention theory, suicide intervention theory, and theories related to the development and change of college students' psychological personalities [20]. At present, many scholars have studied the construction of the psychological crisis intervention system for college students, but due to the late start of domestic research, there are still some differences on many issues, and there is no set of perfect and operable intervention system for college students' psychological crisis.

## 3. Theoretical Definition of Psychological Crisis

### 3.1. Definition of Psychological Crisis

Webster's Dictionary defines a crisis as “a decisive or critical time, phase, or event.” The dictionary defines “crisis is a state of tension.” In Chinese, the literal meaning of the word crisis means “danger,” and it also contains “opportunity.”

Thus, a psychological crisis emphasizes the enormous impact of a crisis event on the human psyche, which is essentially a state of the psychological imbalance that occurs with the occurrence of a crisis event. The inevitability of a crisis event in the development of an individual determines that a psychological crisis is inevitable. In a crisis state, individuals will experience a series of negative emotions as well as physiological, cognitive, and behavioral reactions, and if the crisis reactions are not relieved in time, they will trigger the generation of physiological and psychological disorders. Therefore, it is important to initiate a psychological crisis intervention system for these individuals to prevent these disorders before they are triggered.

### 3.2. Classification of Psychological Crises

There are many classifications of psychological crises, and the more popular one is the trichotomy proposed by psychologist Brammer, namely, developmental crisis, situational crisis, and existential crisis. Developmental crises are abnormal reactions caused by rapid changes in the course of normal growth and development of the individual.

College students are in a special developmental period of their lives, full of desire and enthusiasm for exploration and knowledge, but due to their physical maturity but late psychological maturity, when they encounter a major personal event and are unable to regulate and control their emotions and behaviors, they will experience serious psychological imbalance, and thus, their psychological state will inevitably be in a state of crisis. However, the same event does not necessarily cause a psychological crisis for everyone because major events and traumas do not constitute a crisis in themselves, but only when individuals perceive them as a threat to the satisfaction of their individual needs, their own safety, or their meaningful existence, resulting in their internal imbalance, which leads to a psychological crisis. There are three factors that influence whether an event can be transformed into a psychological crisis for college students: first, the individual's definition of the event and the perception of the impact of the event on him or her; second, whether the individual has a social support system that can give him or her effective help in time; third, whether the individual is provided with effective coping mechanisms, i.e., effective ways to solve problems from past experiences, such as confiding in others, crying, and anger. Because individuals vary greatly in these three areas, the same event may not constitute a psychological crisis for everyone.

### 3.3. Characteristics of College Students' Psychological Crisis

College students are the valuable human resource wealth of society, but the current mental health condition of college students is not optimistic, and the impact of the psychological crisis on college students' mental health cannot be ignored. At the same time, the psychological crisis of college students is characterized by development, interaction, susceptibility, and potentiality.

The successful transition of each psychological crisis is a step towards the maturity and perfection of college students' psychology. Recognizing the characteristics of college students' psychological crisis undoubtedly provides favorable conditions for constructing college students' psychological crisis intervention system and overcomes the blindness, which becomes the entry point and direct basis for concrete practice.

## 4. Research Methodology

### 4.1. Text Preprocessing

In this study, 8501 microblogs were preprocessed by text splitting. Based on the feature that @ users of microblogs automatically add spaces after their user names, the content between the “@” symbol and the first space after it is considered to be the user's @ content, and this part of the text has no practical meaning, so it should be deleted. In addition, since the names of film and television or literary works are often not consistent with their contents, which may be misleading to semantic judgment, the content in the book title number “The” is deleted. Since the frequency of English in blog posts is too small to be analyzed, and the text also contains some special symbols or meaningless words (e.g., and, ah) and URLs that are difficult to extract information, the text is filtered and only characters with Unicode between 4E00 and 9FFF are retained. Then, we used the jieba word splitting package to split the words in the Weibo blog posts and finally removed the words that contained less information (e.g., ah, hey, right). After filtering, 126 nonsuicidal tweets were filtered out, and 880 suicidal tweets and 7221 nonsuicidal tweets were retained as subjects [21, 22].

### 4.2. Eigenvalue Extraction

In this study, the cardinality test is used to extract the eigenvalues. The larger the chi-square value, the more it does not match; the smaller the chi-square value, the smaller the deviation, the more it tends to match, and if the two values are exactly equal, the chi-square value is 0, indicating that the theoretical value is exactly the same. We want to extract the words that are closely related to “suicide,” so for each word, we take the original hypothesis as the word is independent of “suicide” and then calculate the chi-square statistic. The higher the value of the chi-square statistic, the higher the rejection of the hypothesis that the word is related to “suicide.” First, we counted the total number of tweets *N* in the study data, the number of “suicidal” tweets *A*, the number of “nonsuicidal” tweets *B*, the number of “suicidal” tweets *C*, and the number of “non-suicidal” tweets *D* that did not appear. Then, the cardinality value *N*(AD − BC)^2^/(*A*+*C*)(*A*+*B*)(*B*+*D*)(*B*+*C*) was calculated and the one with the higher cardinality value among all the words was selected as the characteristic word [23, 24].

After the feature words were selected, the TF − IDF value of each feature word was calculated for each post, and this value was used as the weight of the feature word, and the data sample was analyzed by principal component analysis. At this point, a microblog can be mapped to a feature vector.

Considering the diversity of Chinese words and to ensure the effectiveness of the prediction model, the first *N*(*N*=2000) words are selected as feature words in this study, which are the feature dimensions in the subsequent model training.

### 4.3. MLP Modeling

This study uses the *Python* deep learning library Theano to implement the modeling process of multilayer perceptron (MLP)-based deep learning algorithms. MLP (multilayer perceptron) neural network is a common ANN algorithm, which consists of an input layer, an output layer, and one or more hidden layers. The model of binary classification perceptron in MLP is shown in Figure 1; *f* is the threshold function: *y*=*f*(∑_*i*=1_^*n*^*w*_*i*_*x*_*i*_+*θ*), which can also be expressed as *y*=sgn(∑_*i*=1_^*n*^*w*_*i*_*x*_*i*_+*θ*), set the threshold value: *θ*=−*w*_0_,  *W*=(*w*_1_, *w*_2_,…,*w*_*n*_, *w*_0_)^*T*^,  *X*=(*x*_1_, *x*_2_, ..., *x*_*n*_, 1)^*T*^. Then, *y*=sgn(*W*^*T*^*X*), that is, $y=f\left(W^{T}X\right)=\left\{\begin{array}{c} 1\;W^{T}X>0\\ -1\;W^{T}X<0 \end{array}\right.\Rightarrow X\in \left\{\begin{array}{c} \omega_{i}\\ \omega_{i} \end{array}\right.$. This neuron has no internal state transitions, and the function is thresholded, so it is actually a linear threshold computational unit. The algorithm of the perceptron is to “learn” the coefficients of the discriminant function from the training sample data set. When training with sample data, if *X* ∈ *ω*_*i*_ and *g*(*X*) > 0, then *W* remains unchanged. If *g*(*X*) < 0, then *W* is modified until all samples satisfy the condition. With the above definition, the perceptron problem becomes *ω*_*i*_/*ω*_*j*_ a two-class problem. Therefore, the idea of self-organization and self-learning of perceptrons can be used for the training of deterministic classifiers. In this study, we build two types of classifiers for “suicidal” and “not suicidal” to predict the suicidal intention of microblog users [25–27].

In order to select the most effective number of hidden nodes, a total of 19 hidden nodes, 50, 100, 150, 200, ..., 950, are chosen to verify the convergence and the corresponding prediction error rate. The basic parameters used in the model are shown in Table 1.

As can be seen from Table 1, for parameter Learning_rate, the value is 0.01; for L1_ Reg transition fitting, the value is 0.01; for L2_ Reg transition fitting, the value is 0.0049; for *n*_ epochs maximum convergence times, the value is 320; for Batch _size batch number, the value 55; for *n*_hidden node number of the best hidden layer, the value is 560; for N_ features dimension (2000 keywords), the value is 2000; for *n*_output number of categories (two categories, suicide and nonsuicide), the value is 2.

### 4.4. Model Validation

In this study, the collected microblogging data were randomly divided into 2 groups, the first group of 70% training data set for MLP model training and modeling and the second group of 30% test data set for testing and validating the accuracy of prediction using the established MLP model.

### 4.5. Statistical Analysis

In order to verify the validity of the eigenvalues and their weights identified by the model, this study used SPSS 19.0 software to analyze the differences between groups in the number of extracted eigenvalues and the corresponding weights [28, 29].

First, the data were analyzed by using the independent sample *t*-test for those samples that were normally distributed and the Mann–Whitney U rank sum test for those that were not normally distributed. Considering the large sample size of this study, Excel was used to calculate the effect size (Cohen's d) based on the analysis of variance in order to avoid the error caused by the data size. The effect size is an indicator of the strength of association between the independent and dependent variables that does not depend on the sample size.

## 5. Results and Analysis

### 5.1. Validation of MLP Model Effect

The prediction results of the MLP model show that the accuracy of the model can reach more than 94%. As shown in Figure 2, the number of nodes ranges from 50 to 950, and the error is around 6%. Considering the convergence effect of the model and the corresponding execution efficiency, this experiment suggests using 550 as the effective number of hidden nodes for the model.

### 5.2. Statistical Results

The process of MLP model training is the process of training and learning the eigenvalues, so the extraction of the eigenvalues has an important impact on the accuracy of the model. In order to verify the effectiveness of the extracted eigenvalues in this study, statistical methods were adopted to analyze the variance of the extracted eigenvalues and their corresponding weighting coefficients.

The results of the K–S test showed that the number of eigenvalues and their corresponding weight values did not conform to a normal distribution (*P* < 0.05), and thus, the Mann–Whitney U rank sum test was performed on the number of eigenvalues and their corresponding weight values of the two groups of data. The results showed that the differences between the number of eigenvalues, and their corresponding weights were statistically significant (*P* < 0.05) (see Table 2).

The results of the effector calculation show (see Table 3) that the difference effect between the number of eigenvalues and their corresponding weight values is large, where the difference effect of the eigenvalue weight values is better than that of the number of eigenvalues, which is a better indication that the eigenvalues and their weights used in the model have a good predictive effect.

### 5.3. Comparison with Other Algorithms

There are many methods for text classification, such as Bayesian, K-nearest neighbor, support vector machine, decision tree, and neural network, and each of these algorithms has its own advantages. Of course, these classification algorithms are also applicable to Chinese text classification. However, considering that the data studied in this experiment are massive and diverse microblog data, and the purpose of this experiment is to suggest an effective suicide intention recognizer, the model needs to have a higher accuracy and better stability.

In this experiment, two methods, plain Bayesian and random forest, are chosen to compare with the MLP multilayer neural network method selected for the experiment to verify that the model implemented by MLP can have better prediction of suicidal intention. The Plain Bayesian algorithm is an algorithm based on Bayesian correlation theory, a probabilistic model-based approach that presupposes mutual independence between attributes given a target value. The random forest algorithm is derived from the machine learning of decision trees, which is a classifier containing multiple decision trees. The training of a decision tree is the process of splitting a data set into two sub-data sets. The training of a neural network is a feature vector as input, passing that vector to the hidden layer, then calculating the result by weight and excitation function, and passing the result to the next layer until finally passed to the output layer before the classification is finished, which is a highly complex nonlinear dynamical system. As shown in Table 4, the prediction error rate of the plain Bayesian algorithm using Weka is 9.17% and the prediction error rate of the random forest algorithm is 8.89%, which shows that the MLP multilayer neural network based on the jieba disambiguation and TF-IDF feature extraction is the most effective prediction model.

## 6. Conclusion

In this paper, we proposed a text analysis-based approach to implement the MLP two-class classifier to achieve automatic recognition and classification of suicide risk based on microblogs. The validity of jieba disambiguation and TF − IDF feature extraction was verified by statistical analysis, and the comparison with other two algorithms verified that MLP has a higher recognition accuracy.

With the development of social networks in recent years, there are more and more people expressing suicidal thoughts on online platforms, and even live-streaming suicide. Therefore, identifying the suicidal intention of users on social networks will become an effective means of suicide prevention. Limited by the data resources and level, the work in this paper needs further improvement. Considering the diversity of Chinese speech, future work will consider additional data resources and better algorithms for eigenvalue extraction, and further research will also consider more demographic factors related to suicide to make suicide prediction more effective.

## Figures and Tables

**Figure 1:** Perception with two classifiers.

**Figure 2:** Iteration number and validation errors for different hidden layer nodes.

**Table 1:** Parameter setting.

Parameter	Value
Learning_rate	0.01
L1_ reg transition fitting	0.001
L2_ reg transition fitting	0.00049
*n*_ epochs maximum convergence times	320
Batch_size batch number	55
n_hidden node number of the best hidden layer	560
N_ features dimension (2000 keywords)	2000
n_output number of categories (two categories, suicide and nonsuicide)	2

**Table 2:** Rank sum test results of key word number and weighting.

Project	Suicidal intention group (*n* = 666)		No suicidal intention group (*n* = 6551)		U value	*W* value	Z value	*P* value
	*M*	*n*	*M*	*n*				
Eigenvalue quantity	7.899	666	4.701	6551	1497001.61	22925001.49	−12.99	0.0001
Eigenvalue weight	54.112	666	17.801	6551	863112.02	22289997.51	−24.98	0.0001

**Table 3:** Results of Cohen's d.

Project	Cohen's d
Eigenvalue quantity	0.949
Eigenvalue weight	1.970

**Table 4:** Validation error comparison among three algorithms %.

Algorithm	Error rate (%)
Naive Bayes	9.17
Random forest	8.89
Multilayer neural networks (MLP)	6.50

## Data Availability

The data set used in this paper is available from the corresponding author upon request.

## References

[1] Waters L. (2011). A review of school-based positive psychology interventions. *Australian Educational and Developmental Psychologist*.

[2] Yao F., Zhang A. (2021). Integration of education management and mental health in psychological crisis intervention in colleges and universities. *ASP Transactions on Psychology and Education*.

[3] Yusoff Y. M. (2012). Self-efficacy, perceived social support, and psychological adjustment in international undergraduate students in a public higher education institution in Malaysia. *Journal of Studies in International Education*.

[4] Ghane Sangatash A., Mirzazadeh Z. S., Azimzadeh S. M., Abdolmaleki H. (2016). The role of psychological capital on social capital of Physical Education Students of Mashhad Universities. *Applied Research in Sport Management*.

[5] Cogenli M. Z., Barli O. (2013). The exposure of psychological violence (mobbing) in universities and an application to the academicians. *Procedia—Social and Behavioral Sciences*.

[6] Lamentan A. M., Yuen C. F. (2020). Psychological empowerment and organisational commitment among academic staff of public universities in Malaysia. *Asian Journal of University Education*.

[7] Zell M. C. (2010). Achieving a college education: the psychological experiences of Latina/o community college students. *Journal of Hispanic Higher Education*.

[8] Kolesnikov A. A., Danilenko I. A., Zimovets N. V. (2019). Social and psychological features of inter-cultural adaptation of Russian students in different universities. *Cypriot Journal of Educational Sciences*.

[9] Kibret B. T., Tareke G. (2017). The contribution of instructor, peer and university support for promoting psychological well-being among students in the Amhara Regional universities. *Clinical and Experimental Psychology*.

[10] Jury M., Smeding A., Stephens N. M., Nelson J. E., Aelenei C., Darnon C. (2017). The experience of low-SES students in higher education: psychological barriers to success and interventions to reduce social-class inequality. *Journal of Social Issues*.

[11] Whitlock J., Prussien K., Pietrusza C. (2015). Predictors of self-injury cessation and subsequent psychological growth: results of a probability sample survey of students in eight universities and colleges. *Child and Adolescent Psychiatry and Mental Health*.

[12] Salami S. O. (2010). Emotional intelligence, self-efficacy, psychological well-being and students attitudes: implications for quality education. *European Journal of Educational Studies*.

[13] Nikpay I., Siadat S., Hoveida R., Nilforooshan P. (2014). A model for investigating the impact of faculty members’ psychological capital on organizational citizenship behaviors in universities. *International Journal of Management Sciences*.

[14] Mugendi S., Githae E. (2021). Relationship between psychological distress and non-completion among postgraduate students in selected public universities in Kenya. *Journal of Humanities and Social Sciences*.

[15] Karimi E., Emadi S. R., Ghanbari S., Nasiri F. (2012). Organizational and psychological wellbeing among western regional universities and their staff. *The Journal of New Thoughts on Education*.

[16] Han L. (2021). Constructing evaluation index system of mental health education in Chinese universities. *ASP Transactions on Psychology and Education*.

[17] Liu P. (2021). Analysis of influencing factors of flip class mode in the application of psychological teaching in colleges and universities. *Recent Advances in Computer Science and Communications*.

[18] Kiyashchuk T. V., Kiyashchuk A. A., Sardarian A. R. (2018). Special aspects of international students’ socio-psychological adaptation at modern universities. *Espacios*.

[19] Cai G., Fang Y., Wen J., Mumtaz S., Song Y., Frascolla V. (2019). Multi-carrier $M$-ary DCSK system with code index modulation: an efficient solution for chaotic communications. *IEEE Journal of Selected Topics in Signal Processing*.

[20] Chandra K., Marcano A. S., Mumtaz S., Prasad R. V., Christiansen H. L. (2018). Unveiling capacity gains in ultradense networks: using mm-wave NOMA. *IEEE Vehicular Technology Magazine*.

[21] Tao X., Zhang C., Xu Y. (2021). Collaborative parameter update based on average variance reduction of historical gradients. *Journal of Electronics and Information Technology*.

[22] Zhengwan Z., Chunjiong Z., Hongbing L. I., Tao X. (2020). Multipath transmission selection algorithm based on immune connectivity model. *Journal of Computer Applications*.

[23] Ibrahim O. K., Romero C., Hassan S., Iqbal M. T. (2022). Mitigating hotspot issues in heterogeneous wireless sensor networks. *Journal of Sensors*.

[24] Ramesh A. K., Alassery F., Kumar A. (2022). Differential evolution algorithm with hierarchical fair competition model. *Intelligent Automation & Soft Computing*.

[25] Zhang Z. W., Wu D., Zhang C. J. (2021). Study of cellular traffic prediction based on multi-channel sparse LSTM[J]. *Computer Science*.

[26] An P., Wang Z., Zhang C. (2022). Ensemble unsupervised autoencoders and Gaussian mixture model for cyberattack detection. *Information Processing & Management*.

[27] Du J., Jiang C., Han Z., Zhang H., Mumtaz S., Ren Y. (2019). Contract mechanism and performance analysis for data transaction in mobile social networks. *IEEE Transactions on Network Science and Engineering*.

[28] Kirko V. I., Malakhova E. V. (2014). Education for the future: new strategies of distance education forthe universities of eastern siberia. *The Turkish Online Journal of Distance Education*.

[29] Hodges L. J., Walker J., Kleiboer A. M. (2011). What is a psychological intervention? A metareview and practical proposal. *Psycho-Oncology*.

